# Ketamine and Propofol Protect Neuron Cells from Oxygen-Glucose Deprivation-Induced Injury through SAPK/JNK Signalling Pathway

This article has been retracted.

**DOI:** 10.1155/2020/8868839

**Published:** 2020-12-15

**Authors:** Aihua Qi, Yiyun Cao, Aizhong Wang

**Affiliations:** Shanghai Jiao Tong University Affiliated Sixth People's Hospital, Shanghai 200233, China

## Abstract

Ketamine and propofol are commonly used anaesthetic reagents. Recent research revealed that ketamine and propofol have an important role in cell survival. However, it remains unknown whether they affect the outcome of hypoxic-ischemic brain injury. To address this issue, we in this study investigated the effects of ketamine and propofol on the survival and proliferation of neuronal PC12 cells after exposure to oxygen-glucose deprivation- (OGD-) induced injury. PC12 cells were maintained under a 3-dimensional (3D) culture system to mimic a real physiological microenvironment. The cell injury was induced by 5% CO_2_ and 95% N_2_ for a different time point. MTT assay was used for the cell proliferation assay. The cell apoptosis was evaluated by annexin V and propidium iodide (PI) labeling, immunofluorescence staining, transmission electron microscopy (TEM), flow cytometry, and Western blot, respectively. Our results showed that PC12 cell apoptosis was significantly increased for up to 70% after the cells were treated with OGD for 24 hours and reduced to baseline at the 72-hour time point. However, pretreatment with ketamine and propofol significantly protected the cells from OGD-induced cell apoptosis, as evidenced by more expression of antiapoptotic Bcl-2 and lower expression of proapoptotic cleaved caspase-3, phosphor-SAPK/JNK, and phosphor-c-Jun than those of untreated control cells. Thus, we conclude that ketamine and propofol protected PC12 cells from OGD-induced cell apoptosis, at least partially through the SAPK/JNK signalling pathway.

## 1. Introduction

Ischemia and hypoxia often occur during surgical operation and can induce severe damage to multiple organs in patients under general anaesthesia. The brain is the mostly affected organ. Severe damage to neuron cells is observed during perioperative hypoxia-ischemia [1, 2]. Thus, it is essential to seek an effective approach in the prevention and treatment of perioperative hypoxic-ischemic brain injury. Ketamine (KTM) and propofol (PPF) are commonly used anaesthesia reagents during surgery [3]. However, recent studies have shown that ketamine and propofol have a protective function in oxygen-glucose deprivation- (OGD-) induced neuron injury [2, 4]. Recent reports suggested that ketamine and propofol may protect microglia against OGD/reoxygenation-induced cell death by binding to Toll-like receptor 4 (TLR4) [5]. It was also reported that propofol can protect endothelial cells during intermittent hypoxia/reoxygenation through suppressing p38MAPK/NF-*κ*B signalling [6].

It is documented that SAPK/JNK signalling is involved in the initiation of neuron cell activation and apoptosis [7, 8]. SAPK/JNK inhibitor SP6000125 successfully reduced cytokine production in low-intensity microwave-exposed RAW 264.7 macrophages [9]. However, little is known about the role and underlying molecular mechanisms of SAPK/JNK signalling in ketamine and propofol-mediated neuron protection. It was documented that the 3-dimensional culture (3D) system mimics the physiological environment much better than the 2-dimensional (2D) culture system. However, it is not well defined whether the 3D system improves neuron cell survival than the 2D system under oxidative stress condition. To address this issue, we in this study maintained neuron cells in both 3D and 2D culture systems. Then, the cells were treated with OGD alone or in conjunction with ketamine and propofol for the indicated time points. Our results revealed a better cell survival and proliferation of neuron cells cultured in the 3D system. In addition, we observed that ketamine and propofol pretreatment significantly improved neuron survival and induced more extended monopolar neurite processes after OGD exposure. The results indicated that the 3D cell culture system is beneficial in promoting neuron cell proliferation, survival, and differentiation. It provided significant molecular bases for the role of ketamine and propofol in preventing OGD-mediated neuron injury and has important implication in the treatment of ischemia and hypoxia during surgical operation.

## 2. Materials and Methods

### 2.1. 3D Cell Culture and Treatment

The PC12 cell line (ATCC, Manassas, VA) was seeded in a 3D system and maintained in RPMI1640 medium supplied with 10% fetal bovine serum (FBS) and nerve growth factor (NGF). Before experimental intervention, the cells were starved in RPMI1640 medium without FBS. The cell injury was induced by maintaining cells in culture medium deficient glucose and under gas containing 0.5% O_2_, 5% CO_2_, and 95% N_2_. The cells were pretreated with 10 mM ketamine and 10 *μ*M propofol 1 minute prior to hypoxic exposure.

### 2.2. Cell Viability Assay

Cell viability was measured by the MTT assay according to the manufacturer instruction. Briefly, the cell supernatants were collected after PC12 cells were exposed to OGD for 0, 6, 12, 24, 48, or 72 hours. Products in cell supernatants were measured by an enzyme-linked immunosorbent assay, and absorbance density (OD) was detected at 570 nm.

### 2.3. Electron Microscopy Analysis

1 × 10^7^ cells were plated on culture dishes. After 10 days of cell culture, the medium was removed, and cells were fixed with 2.5% glutaraldehyde for 2 hours. Then, the cells were washed twice with PBS, dehydrated using ethanol gradient, embedded, solidified, and cut into ultrathin sections. The sections were finally viewed under electron microscopy.

### 2.4. Apoptosis Assay

The cells were digested with 0.2% trypsin to generate a single cell suspension, washed with PBS, and treated with annexin V and PI. The cells undergoing necrosis and apoptosis were visualized under a fluorescence microscope in a blinded manner (5 regions/group) and quantified by flow cytometry.

### 2.5. Western Blot Analysis

Cell lysates were obtained from the treated cells and dissolved in 10% acrylamide/bis gel containing 0.1% SDS. After gel electrophoresis, protein in gels was transferred into nitrocellulose membranes. The blots were incubated with primary antibody and followed by incubation with HRP-conjugated second antibody. After washing with TBST buffer, the blots were developed with ECL substrate solution. Protein bands were quantified using densitometric analysis software (Bio-Rad).

### 2.6. Statistical Analysis

All data was presented as means ± sem, and statistical analysis was performed using GraphPad Prism 5 software (GraphPad, USA). A value of *p* < 0.05 was considered statistically significantly different.

## 3. Results

### 3.1. 3D-Matrigel Culture Promoted Neurite Outgrowth of PC12 Cells

Because the current 2D culture system is limited for low efficiency in cell proliferation and differentiation, we in this study cultured neuron cells, PC12, in the 3D system to mimic the cell growth environment in vivo. In parallel culture to the 2D system, we observed more cell growth in the 3D system than in the 2D system, as evidenced by the increased cell number and clusters 48 hours after the cells were cultured in the 3D system, compared to the cells in the 2D system (Figure 1(a)). H&E staining showed the increased monopolar neurites of cells in the 3D system (Figure 1(b)). Therefore, we conclude that the 3D culture system significantly improved neuron cell growth and differentiation.

### 3.2. OGD Induced PC12 Cell Apoptosis That Was Reversed by Pretreatment with Ketamine and Propofol

To investigate the effects of ketamine and propofol on the survival of PC12 cells, we at first established a neuron cell injury model, respectively, in 2D and 3D systems by exposing to OGD. Our results showed that OGD effectively reduced cell viability in a time-dependent manner. However, there was more cell viability cultured in the 3D system than in the 2D system, indicating the beneficial role of the 3D system in neuron cell culture (Figure 2(a)). Further electron microscopy showed that OGD treatment resulted in lower growth of cell neurites (Figure 2(b)) and induced more cell shrinkage, indicative of cell apoptosis (Figure 2(c)).

To further define whether ketamine (KTM) and propofol (PPF) can reverse OGD-induced cell apoptosis, we pretreated the neuron cells with ketamine or propofol prior to OGD exposure. The results showed that ketamine or propofol pretreatment effectively suppressed the OGD-induced annexin V+PI+ apoptotic cells (Figure 3(a)). There was around 2-fold reduction of apoptotic cells pretreated with ketamine or propofol, compared to the OGD treatment alone (Figure 3(b), *p* < 0.05 and *p* < 0.01, *n* = 3). Accordingly, the cell viability was significantly increased in the ketamine (Figure 3(c))- and propofol (Figure 3(d))- pretreated cells under a concentration-dependent manner, compared to the untreated cells. Consistent with the finding in Figure 2(a), we also observed better cell viability in the 3D system than in the 2D system when the cells were pretreated with ketamine and propofol. Thus, ketamine and propofol were beneficial in preventing OGD-induced neuron cell apoptosis in vitro.

### 3.3. Pretreatment with Ketamine and Propofol Reduced the Expression of p-SAPK/JNK and Cleaved Caspase-3 in PC12 Cells

Whether the reduced cell apoptosis by ketamine or propofol pretreatment is associated with the altered expression of apoptosis relevant molecules was further investigated. Our further analysis by Western blot showed that OGD significantly increased the expression of p-SAPK/JNK and p-c-Jun. However, pretreatment with ketamine and propofol effectively reversed the OGD-induced upregulation of p-SAPK/JNK and p-c-Jun (Figures 4(a) and 4(b)). In addition, we observed the increased expression of apoptotic cleaved caspase-3 but reduced expression of antiapoptotic Bcl-2 in the OGD-treated cells. However, ketamine and propofol pretreatment effectively reversed the altered expression of cleaved caspase-3 and Bcl-2 (Figures 4(c) and 4(d)). The results were also further confirmed by immunostaining analysis, in which ketamine and propofol pretreatment significantly reversed the OGD-induced upregulation of cleaved caspase-3 in the neuron cells (Figure 4(e)). Therefore, ketamine and propofol both exerted antiapoptotic function through the SAPK/JNK signalling pathway in the OGD-treated neuron cells.

## 4. Discussion

Hypoxemia is a common cause of acute neuron injury. In the injured neuron area, massive inflammation and a large amount of proinflammatory cytokines are expressed, due to hypoxemia-induced oxidative stress and cell damage [10, 11]. Treatment with anti-inflammatory reagents and neurotrophic factors becomes essential in the prevention and treatment of acute neuron injury in vivo [10, 12]. Because it was previously reported that 3D in vitro culture promoted more efficient neuronal differentiation of stem cells, inducing more peripheral nerve regeneration than 2D in vitro culture [13], we in this study compared neuron cell growth in the 3D system and 2D system. After 3 days in culture, we observed higher cell growth and viability in the 3D cell culture system than the 2D cell culture system. In addition, more monopolar neurites were observed in the 3D system, indicating the beneficial role of the 3D culture model in improving neuron proliferation and differentiation.

By using this system, we further investigated the effects of ketamine and propofol in OGD-induced neuron injury. Our results showed that OGD can effectively induce acute neuron cell injury, as indicated by the higher number of cell apoptosis and lower cell survival starting 6 hours after OGD exposure. However, we observed a significantly reduced neuron cell apoptosis and death after neuron cells were cotreated with both OGD and ketamine or propofol, compared to the cells treated with OGD alone. The results indicated the therapeutic role of ketamine and propofol in suppressing hypoxemia-induced neuron cell injury. Ketamine and propofol are commonly used anaesthesia reagents in clinical practice. Recent study revealed that both ketamine and propofol have anti-inflammatory function in glial cells [14, 15]. Based on our results, ketamine and propofol should be considered promising adjuvants in the treatment of hypoxemia-induced acute neuron injury and suppressing local inflammation. More studies in the animal model will be performed to define their therapeutic benefits in the future.

However, it is still not clear how ketamine and propofol exert anti-inflammatory function and promote neuron survival in this study. Previously reported results showed that ketamine and propofol can suppress LPS-induced upregulation of IL-1beta and extracellular signal-regulated kinase 1/2 (ERK1/2) phosphorylation in glia cells and brains [15, 16]. IL-1beta is a proinflammatory cytokine and critically participates in cell activation and death of macrophage pyroptosis [17, 18]. TNF-alpha, tumor necrosis factor-related apoptosis-inducing ligand (TRAIL), and IFN-gamma are a potent inducer of neuron, microglia, and astroglia apoptosis after hypoxia-ischemia and inflammation [1, 19]. However, inhibition of the JAK/STAT1 pathway in IFN-gamma-injected animals effectively reduced microglial activation and microglia-mediated neuroinflammation and neurogenic injury [20]. The results displayed the critical role of these cytokines in neuronal inflammation and injury. Ketamine and propofol may protect neuron cells from oxidative stress-induced injury through suppressing these signalling pathways and production of proinflammatory cytokines.

Our further study in vitro also revealed the increased activation of SAPK/JNK signalling in the OGD-treated neuron cells, but the activated SAPK/JNK signalling was significantly suppressed in the OGD/ketamine- or OGD/propofol-cotreated cells, indicating the involvement of SAPK/JNK signalling in ketamine and propofol-mediated neuron survival. It was previously reported that SAPK/JNK signalling was critically involved in cell activation and apoptosis under oxidative stress, because SAPK/JNK inhibitor SP600125 can reverse porcine epidemic diarrhea virus-induced Vero cell apoptosis [8]. In addition, SP6000125 treatment can effectively suppress cytokine production in low-intensity microwave-exposed macrophages. These results indicated the important role of SAPK/JNK signalling in cell activation, apoptosis, and inflammation [9]. Therefore, SAPK/JNK signalling was associated with neuron activation and apoptosis. Ketamine and propofol may prevent neuron cells from OGD-induced acute injury and neuron cell apoptosis through suppressing the SAPK/JNK signalling pathway.

In summary, the results indicated that 3D culture significantly improved neuron cell growth and survival. Ketamine and propofol exerted significant activities against OGD-induced neuron cell injury. The protective effects are at least partially associated with suppressing the SAPK/JNK signalling pathway. Therefore, ketamine and propofol not only induced anaesthesia and sedation but also had neuroprotective effects.

## Figures and Tables

**Figure 1:** 3D-matrigel culture promoted neurite outgrowth of PC12 cells. (a) PC12 neuron cells were cultured in 2D and 3D culture systems, respectively, for 24 hrs and 48 hrs. The pictures were taken under a contrast microscope at a magnification of 200x. (b) Representative H&E staining of PC12 cells cultured in the 3D system. Representative photograph was shown.

**Figure 2:** OGD induced PC12 cell apoptosis. (a) PC12 cells cultured in 2D and 3D systems were exposed to OGD for a different time point. The cell viability was measured by MTT assay. Data was presented as the mean ± standard error, *n* = 3. ^∗^*p* < 0.05 vs. the cells at 0 time point. (b) PC12 cells cultured in the 3D system were treated with OGD or untreated for 48 hrs, and the cell morphology was identified by an electron microscope at magnification of 200x, 1500x, and 5000x. The OGD-treated cells had low neurite growth. (c) The apoptotic PC12 cells under an electron microscope. Representative photograph was shown.

**Figure 3:** Ketamine and propofol pretreatment improved the PC12 cell survival and suppressed cell apoptosis. PC12 cells cultured in 2D and 3D systems were pretreated with different concentrations of ketamine (KTM) (a) and propofol (PPF) (b) for 1 minute before OGD exposure. The treated cells were analyzed for cell viability by MTT at 48 hours after OGD exposure. Data was presented as the mean ± standard error, *n* = 3. ^#^*p* < 0.05 vs. the cells treated with 0/OGD, ^∗^*p* < 0.05 vs. the cells cultured in the 2D system. (c) The cells were pretreated with 10 mM ketamine and 10 *μ*M propofol 1 minute before RGD treatment for 48 hours. Flow cytometry analysis for apoptotic cells. The annexin V+ cells were identified as apoptotic cells. One representative dot plot of three independent experiments was shown. (d) Quantitative analysis of apoptotic cells in the treated cells. ^∗^*p* < 0.05, ^∗∗^*p* < 0.01 vs. the cells treated with 0/OGD, *n* = 3.

**Figure 4:** Pretreatment with ketamine and propofol reduced the expression of p-SAPK/JNK and cleaved caspase-3 in PC12 cells. (a) The expression of p-SAPK/JNK and p-Jun in the treated cells was analyzed by Western blot analysis. One representative blot was shown. (b) Quantitative analysis of p-SAPK/JNK and p-Jun expression in the treated cells by ImageJ software; data was presented as the ratio of phosphorylated protein to total protein in each lane. (c) Representative blot for the expression of caspase-3 and Bcl-2 in the treated cells; (d) quantitative analysis of the cleaved caspase-3 and Bcl-2 expression by ImageJ software. Data was presented as the ratio of cleaved caspase-3 to procaspase-3, or the ratio of Bcl-2 to internal control GAPDH in each lane. *n* = 3. ^∗^*p* < 0.05, ^∗∗^*p* < 0.01 vs. the cells treated with 0/OGD control. (e) The expression of cleaved caspase-3 in the treated cells was detected by immunostaining. The positive cells were quantitatively analyzed, and data was presented as the mean number of cleaved caspase-3+ cells per field ± standard error. *n* = 6 field/treatment.

## Data Availability

All data, models, and code generated or used during the study appear in the submitted article.
